# Early cartilage abnormalities at the hip are associated with obesity and body composition measures – a 3.0T MRI community-based study

**DOI:** 10.1186/s13075-015-0618-1

**Published:** 2015-04-22

**Authors:** Andrew J Teichtahl, Yuanyuan Wang, Sam Smith, Anita E Wluka, Donna Urquhart, Graham G Giles, Sultana Monira Hussain, Flavia M Cicuttini

**Affiliations:** Department of Epidemiology and Preventive Medicine, School of Public Health and Preventive Medicine, Monash University, Alfred Hospital, Melbourne, VIC 3004 Australia; Baker IDI Heart and Diabetes Institute, Commercial Road, Melbourne, VIC 3004 Australia; Centre for Epidemiology and Biostatistics, Melbourne School of Population and Global Health, The University of Melbourne, Carlton, VIC 3053 Australia; Cancer Epidemiology Centre, Cancer Council Victoria, Melbourne, VIC 3004 Australia

## Abstract

**Introduction:**

Although obesity is a risk factor for hip osteoarthritis (OA), the role of body composition, if any, is unclear. This study examines whether the body mass index (BMI) and body composition are associated with hip cartilage changes using magnetic resonance imaging (MRI) in community-based adults.

**Methods:**

141 community-based participants with no clinical hip disease, including OA, had BMI and body composition (fat mass and fat free mass) measured at baseline (1990 to 1994), and BMI measured and 3.0 T MRI performed at follow-up (2009–2010). Femoral head cartilage volume was measured and femoral head cartilage defects were scored in the different hip regions.

**Results:**

For females, baseline BMI (β = −26 mm^3^, 95% Confidence interval (CI) -47 to −6 mm^3^, p = 0.01) and fat mass (β = −11 mm^3^, 95% CI −21 to −1 mm^3^, p = 0.03) were negatively associated with femoral head cartilage volume. Also, while increased baseline fat mass was associated with an increased risk of cartilage defects in the central superolateral region of the femoral head (Odds Ratio (OR) = 1.08, 95% CI 1.00–1.15, p = 0.04), increased baseline fat free mass was associated with a reduced risk of cartilage defects in this region (OR = 0.82, 95% CI 0.67–0.99; p = 0.04). For males, baseline fat free mass was associated with increased femoral head cartilage volume (β = 40 mm^3^, 95% CI 6 to 74 mm^3^, p = 0.02).

**Conclusions:**

Increased fat mass was associated with adverse hip cartilage changes for females, while increased fat free mass was associated with beneficial cartilage changes for both genders. Further work is required to determine whether modifying body composition alters the development of hip OA.

## Introduction

Osteoarthritis (OA) of the hip and knee are common and painful conditions that often require costly joint replacement surgery for end-stage disease. Most studies examining the pathogenesis of OA have focussed on cartilage as the primary endpoint, predominantly via examining radiographic joint space width as an indirect measure of articular cartilage. It is now well-recognised that radiographic joint space narrowing is a relatively late sign of hip OA, with a 13% mean reduction in femoral head cartilage volume occurring by the time the first changes in radiographic joint space narrowing become present [1].

With the advent of magnetic resonance imaging (MRI), it is possible to directly examine articular cartilage. Cartilage defects represent localised cartilage pathology and predict pain, cartilage volume loss and joint replacement surgery at the knee [2-4]. Cartilage defects are not as well-studied at the hip, but have been associated with self-reported pain, disability and radiographic OA [5,6]. By examining risk factors that are associated with early structural hip changes such as reduced cartilage volume and the presence of cartilage defects, it may be possible to better understand early pathological processes and develop interventions that aim to avert or delay the development and/or progression of hip OA.

Although obesity is the major modifiable risk factor for knee OA [7-9], the relationship between obesity and hip OA is less consistent [10-15]. The most commonly employed measure of obesity is the body mass index (BMI), which has been shown to predict hip replacement [16] but BMI fails to account for body composition and cannot discriminate adipose from non-adipose body mass [17]. At the knee, body composition studies have shown a detrimental effect of fat mass and a beneficial effect of fat-free mass on knee cartilage [18-20], with a recent systematic review concluding that fat mass is associated with the early structural changes of cartilage defects [21]. At the hip, adiposity measures such as fat mass have been shown to be associated with an increased risk of hip joint replacement [16] but there are no data available to examine whether body composition is associated with structural changes at the hip.

The aim of this study was to examine associations between BMI and body composition (fat and fat-free mass) and femoral head cartilage volume and defects in community-based adults with no diagnosed hip OA.

## Methods

### Participants

One hundred and forty-one people with no diagnosed hip OA were recruited between 2009 and 2010 from the Melbourne Collaborative Cohort Study (MCCS), a prospective cohort study of residents of Melbourne, Australia, aged 40 to 69 years at MCCS inception (1990 to 1994) [22]. Participants were eligible for the current study if they were aged 50 to 85 years without any of the following exclusion criteria: a medical or allied health professional diagnosis of hip OA; significant hip pain lasting for >24 hours in the last 5 years; a previous hip injury requiring non weight-bearing treatment for >24 hours or surgery (including arthroscopy); or a history of any form of arthritis diagnosed by a medical practitioner. Participants were further excluded if they had any malignancy or any contraindication to MRI, including a pacemaker, metal sutures, presence of shrapnel or iron filings in the eye, or claustrophobia. The study was approved by the Human Research Ethics Committees of The Cancer Council Victoria and Monash University. All participants gave written informed consent.

### Anthropometric data

Height and weight were measured at baseline assessment during 1990 to 1994 and repeated at the time of hip MRI during 2009 to 2010. Weight was measured to the nearest 100 g using digital electronic scales. Height was measured to the nearest 1 mm using a stadiometer. BMI was calculated as the weight in kilograms divided by the square of height in meters.

### Body composition measures

Bioelectric impedance analysis was performed at baseline (1990 to 1994) with a single-frequency (50 kHz) electric current produced by a BIA-101A RJL system analyser (RJL systems, Detroit, MI, USA) during 1990 to 1994. Resistance and reactance were measured with subjects in the supine position. The non-adipose mass, hereafter termed fat-free mass, was estimated [23] in male subjects as:

9.1536 + (0.4273 × Height^2^/Resistance) + (0.1926 × Weight) + (0.0667 × Reactance).

Fat-free mass in female subjects was estimated as:

7.7435 + (0.4542 × Height^2^/Resistance) + (0.119 × Weight) + (0.0455 × Reactance).

The adipose mass, hereafter termed fat mass (FM). FM was calculated as:

FM = Weight – Fat-free mass.

Body-fat percentage was calculated by dividing FM by weight and multiplying by 100.

### MRI measurements

Each participant had MRI performed on their dominant hip, defined by the leg used to kick a ball (89% right sided), during 2009 to 2010, an average of 16.9 (±0.61) years after MCCS inception. Hips were imaged on a 3.0-T whole body magnetic resonance unit (Siemens, Verio, Siemens Medical, Germany) using a phased array flex coil. Sagittal images were obtained using a T_2_-weighted fat-suppressed three-dimensional gradient-recalled acquisition sequence in the steady state (repetition time 14.45 msec, echo time 5.17 msec; flip angle 25°, slice thickness 1.5 mm, field of view 16 cm, pixel matrix 320 × 320, acquisition time 7 minutes 47 seconds, and one acquisition). Coronal images were obtained using a fat saturation, proton density, spin-echo acquisition sequence (repetition time 3,400 msec, echo time 64 msec, flip angle 90°, slice thickness 3 mm, field of view 16 cm, pixel matrix 256 × 256, acquisition time 5 minutes 26 sec, and one acquisition).

Femoral head cartilage volume was measured from T_2_-weighted sagittal images using the software Osiris (version 4.19; Geneva University Hospital, Geneva, Switzerland) as previously described [1]. The image data were transferred to the workstation, and an isotropic voxel size was then obtained by a trilinear interpolation routine. The volume of the femoral head cartilage was isolated from the total volume by drawing disarticulation contours around the cartilage boundaries on each image section. These data were then resampled by bilinear and cubic interpolation for the final three-dimensional rendering. The volume of the femoral head cartilage was determined by summing all the pertinent voxels within the resultant binary volume. Femoral head cartilage volume was measured in duplicate with at least a one-week interval by one trained observer. The coefficient of variation (CV) was 2.5% [1]. The intra-observer reproducibility (assessed by intra-class correlation coefficient, ICC) was 0.99.

The femoral head was divided into three regions: central, anterior and femoral to assess cartilage defects. The anterior and posterior regions were assessed in the sagittal plane and corresponded to the first and last three coronal slices (9 mm) (Figure 1A). The area in between the anterior and posterior region was termed the central region. Femoral head cartilage defects were assessed from proton density coronal images and confirmed on sagittal imaging for the central region, and from the sagittal imaging for the anterior and posterior regions. The presence of cartilage defects was defined as loss of cartilage thickness of more than 50% which was shown on at least two consecutive slices. One trained observer, who was blinded to participants’ characteristics, assessed the presence of cartilage defects for each participant in duplicate, at least one week apart. The intra-observer reproducibility (ICC) was 0.72. The central region was further subdivided in the coronal plane (Figure 1B). The intersection of the axis of the femoral head and neck was considered to be the midpoint of the region, with the axis of the femoral neck used to demarcate the central superolateral from the central inferomedial region. The division of anterior, central and posterior regions was adapted from methods used in previously published works [5,6].

**Figure 1:** Regional zones of the hip joint. **(A)** Sagittal image depicting the anterior, central and posterior regions. **(B)** Coronal image depicting the central superolateral (CSL) and inferomedial (CIM) regions.

The sagittal image closest to the centre of the femoral head was used to measure the femoral head bone area. It was measured by drawing contours around the femoral head bone, and the area was calculated automatically by the Osiris program as an indicator of bone size. Femoral head bone area was measured by one trained observer with 50 random cross-checks performed by a second observer. The CV was 1.1% [1]. The inter-observer reproducibility (ICC) was 0.99.

### Statistical analyses

Multiple linear regression analyses were used to determine the relationships between obesity and body composition measures with femoral head cartilage volume. Binary logistic regression was used to determine the relationships between femoral head cartilage defects and BMI and body composition measures. Because body composition and femoral head cartilage volume differed significantly between men and women, genders were examined separately, with adjustments for age, femoral head bone area and another marker of body composition. For instance, when fat mass was the independent variable, fat-free mass was adjusted for in multivariate analyses. In contrast, when fat-free mass was the independent variable, fat mass was adjusted for in multivariate analyses. To examine whether there was multicolinearity between fat-free mass and fat mass, we performed a colinearity diagnosis. In men, the Pearson correlation between fat-free mass and fat mass was 0.39, with the tolerance of 0.80 for both fat-free mass and fat mass. In women, the Pearson correlation was 0.40, with the tolerance of 0.68 for fat-free mass and 0.78 for fat mass. Therefore, there was no multicolinearity between fat-free mass and fat mass and it is appropriate to co-adjust fat mass and fat-free mass in one model. A *P*-value <0.05 (two-tailed) was regarded as statistically significant. All analyses were performed using the SPSS statistical package (standard version 20.0 SPSS, Chicago, IL, USA).

## Results

Subject characteristics are shown in Table 1. Men had greater BMI, femoral head cartilage volume and bone area as well as fat-free mass than women (all *P* <0.01). In contrast, women had greater percentage of body fat than men (37.3% versus 28.8%, *P* <0.001). There was no difference between genders in fat mass or prevalence of femoral head cartilage defects. The prevalence of cartilage defects in the anterior (6.5% versus 1.2%, men to women) and posterior (17.7% versus 17.7%, men to women) region of the femoral head was low for both genders. The median of the total Western Ontario and McMaster University osteoarthritis index (WOMAC) pain score (out of 500) was 19 for men and 22 for women (*P* = 0.36, Mann–Whitney *U*-test).

**Table 1:** **Characteristics of study participants**

	**Men (n = 62)**	**Women (n = 79)**	***P*** ^**1**^
**Baseline measurements (1990 to 1994)**			
Body mass index, kg m^−2^	27.2 (3.5)	25.1 (4.2)	<0.01
Fat mass, kg	24.2 (7.7)	25.0 (8.9)	0.59
Body fat, %	28.8 (6.1)	37.3 (7.0)	<0.001
Fat-free mass, kg	58.3 (5.0)	40.3 (3.6)	<0.001
**Follow-up measurements (2009 to 2010)**			
Age, years	66.2 (6.8)	67.2 (7.8)	0.41
Body mass index, kg m^−2^	28.3 (4.1)	27.0 (5.3)	0.09
WOMAC median pain, out of 500	19	22	-
Femoral head cartilage volume, mm^3^	3891 (636)	2867 (451)	<0.001
Femoral head bone area, mm^2^	1831 (179)	1429 (126)	<0.001
Femoral head cartilage defects, n (%)			
Central superolateral	22 (35.5)	23 (29.1)	0.42^2^
Central inferomedial	30 (48.4)	37 (46.8)	0.86^2^
Anterior	4 (6.3)	1 (1.3)	0.10^2^
Posterior	11 (17.5)	14 (17.7)	0.97^2^

Data presented as mean (standard deviation) or number (%) unless otherwise stated. ^1^ *P*-values represent difference between genders analysed by independent sample *t*-tests unless otherwise stated. ^2^Chi-squared test. WOMAC, Western Ontario and McMaster University osteoarthritis index.

The relationships between BMI and body composition measures and femoral head cartilage volume are shown in Table 2. After adjusting for age and femoral head bone area, BMI at baseline was negatively associated with femoral head cartilage volume in women (β -26 mm^3^, 95% CI −47 to −6 mm^3^, *P* = 0.01), but not men (β 3 mm^3^, 95% CI −37 to 44 mm^3^, *P* = 0.87). That is, for every one unit increase in BMI (kg m^−2^), there was an associated 26 mm^3^ reduction in femoral head cartilage volume in women. BMI at baseline was strongly correlated with BMI at follow up (time of MRI) (*r* = 0.86, *P* <0.0001), while greater BMI at follow up tended toward being associated with reduced femoral head cartilage volume for women (β -15 mm^3^, 95% CI −32 to 1 mm^3^, *P* = 0.06). After adjusting for age, femoral head bone area and fat-free mass, greater fat mass (β -11 mm^3^, 95% CI −21 to −1 mm^3^, *P* = 0.03) and percentage body fat (β -13 mm^3^, 95% CI −26 to −0 mm^3^, p = 0.04) at baseline were both associated with reduced femoral head cartilage volume in women. Fat-free mass at baseline was positively associated with femoral head cartilage volume in men (β 40 mm^3^, 95% CI 6 to 74 mm^3^, *P* = 0.02) but not in women (β 0 mm^3^, 95% CI −29 to 29 mm^3^, *P* = 0.98) after adjustment for age, femoral head bone area and fat mass.

**Table 2:** **Associations between baseline obesity and body composition measures and femoral head cartilage volume (mm** ^**3**^ **)**

	**Men**				**Women**			
	**Univariate regression β**	***P***	**Multivariate regression β**	***P***	**Univariate regression β**	***P***	**Multivariate regression β**	***P***
	**(95% CI)**		**(95% CI)**		**(95% CI)**		**(95% CI)**	
**1990 to 1994**								
BMI^1^, kg m^−2^	1 (−47, 49)	0.96	3 (−37, 44)	0.87	−28 (−52, −4)	0.02	−26 (−47, −6)	0.01
Fat-free mass^2^, kg	46 (15, 78)	<0.01	40 (6, 74)	0.02	15 (−14, 43)	0.30	0 (−29, 29)	0.98
Fat mass^3^, kg	13 (−8, 35)	0.22	−3 (−24, 17)	0.73	−8 (−19, 4)	0.17	−11 (−21, −1)	0.03
Body fat^3^, %	4 (−24, 32)	0.78	−6 (−30, 17)	0.60	−13 (−28, 1)	0.08	−13 (−26, 0)	0.04
**2009 to 2010**								
BMI^1^, kg m^−2^	1 (−46, 49)	0.95	9 (−30, 49)	0.65	−22 (−40, −3)	0.03	−15 (−32, 1)	0.06

^1^Adjusted for age and femoral head bone area. ^2^Adjusted for age, femoral head bone area, and fat mass. ^3^Adjusted for age, femoral head bone area and fat-free mass. BMI, body mass index.

The relationships between BMI and body composition measures and femoral head cartilage defects are shown in Table 3. After adjusting for age, femoral head bone area and fat-free mass, increased fat mass at baseline was associated with an increased risk of cartilage defects in the central superolateral region of the femoral head in women (OR 1.08, 95% CI 1.00 to 1.15, *P* = 0.04) but not men (OR 0.99, 95% CI 0.91 to 1.06, *P* = 0.71). Increased fat-free mass at baseline was associated with a reduced risk of prevalent cartilage defects in the central superolateral region of the femoral head in women (OR 0.82, 95% CI 0.67 to 0.99; *P* = 0.04) but not men (OR 1.02, 95% CI 0.93, 1.11, *P* = 0.70) after adjusting for age, femoral head bone area and fat mass. There were no significant associations between BMI and femoral head cartilage defects, or between body composition measures and cartilage defects in the central inferomedial region of the femoral head. The low prevalence of cartilage defects at the anterior femoral head in this cohort precluded analyses for this region, and there was no significant associations found for cartilage defects at the posterior femoral head (data not shown).

**Table 3:** **Associations between baseline obesity and body composition measures and femoral head cartilage defects**

	**Men**				**Women**			
	**Univariate odds ratio**	***P***	**Multivariate odds ratio**	***P***	**Univariate odds ratio**	***P***	**Multivariate odds ratio**	**P**
	**(95% CI)**		**(95% CI)**		**(95% CI)**		**(95% CI)**	
**Central superolateral**								
**1990 to 1994**								
Body mass index^1^, kg m^−2^	1.05 (0.91, 1.22)	0.50	1.05 (0.90, 1.22)	0.53	1.09 (0.97, 1.22)	0.14	1.08 (0.96, 1.21)	0.21
Fat-free mass^2^, kg	1.06 (0.95, 1.18)	0.28	1.06 (0.94, 1.20)	0.31	0.93 (0.81, 1.07)	0.32	0.82 (0.67, 0.99)	0.04
Fat mass^3^, kg	1.01 (0.94, 1.08)	0.83	0.99 (0.91, 1.06)	0.71	1.04 (0.99, 1.10)	0.15	1.08 (1.00, 1.15)	0.04
Body fat^3^, %	1.01 (0.93, 1.11)	0.75	1.00 (0.92, 1.10)	0.94	1.07 (0.99, 1.15)	0.07	1.08 (0.99, 1.17)	0.07
**2009 to 2010**								
Body mass index^1^, kg m^−2^	1.02 (0.90, 1.16)	0.76	1.02 (0.90, 1.16)	0.73	1.06 (0.97, 1.16)	0.19	1.07 (0.97, 1.17)	0.18
**Central inferomedial**								
**1990 to 1994**								
Body mass index^1^, kg m^−2^	1.11 (0.95, 1.28)	0.19	1.11 (0.96, 1.29)	0.16	1.00 (0.90, 1.11)	0.96	0.99 (0.88, 1.10)	0.82
Fat-free mass^2^, kg	1.08 (0.97, 1.20)	0.17	1.12 (0.99, 1.27)	0.07	1.00 (0.89, 1.14)	0.97	0.96 (0.83, 1.12)	0.63
Fat mass^3^, kg	0.98 (0.92, 1.03)	0.56	0.96 (0.89, 1.04)	0.35	1.02 (0.97, 1.07)	0.50	1.02 (0.96, 1.08)	0.51
Body fat^3^, %	0.95 (0.87, 1.04)	0.25	0.95 (0.87, 1.04)	0.28	1.03 (0.96, 1.10)	0.40	1.03 (0.96, 1.10)	0.48
**2009 to 2010**								
Body mass index^1^, kg m^−2^	1.13 (0.99, 1.29)	0.08	1.12 (0.98, 1.28)	0.08	1.01 (0.93, 1.10)	0.83	1.01 (0.93, 1.10)	0.80

^1^Adjusted for age and femoral head bone area. ^2^Adjusted for age, femoral head bone area and fat mass. ^3^Adjusted for age, femoral head bone area and fat-free mass.

## Discussion

Increased fat mass was associated with adverse hip cartilage changes in women (reduced cartilage volume and increased cartilage defects), while increased fat-free mass was associated with beneficial cartilage changes in both genders (reduced cartilage defects in the central superolateral region of the femoral head in women; increased femoral head cartilage volume in men). Further work is required to determine whether modifying body composition alters the natural history of hip OA.

This is the first study to directly examine associations between adiposity and hip cartilage volume and defects. A previous systematic review concluded that obesity (measured predominantly by increased BMI) had a moderately positive influence on the development of hip OA, with an odds ratio of approximately two [15]. Nevertheless, previous studies have relied upon radiographic joint space narrowing, an indirect measure of cartilage loss, to assess the relationship between obesity and hip OA [10-15]. In the current study, we measured femoral head cartilage volume from MRI. Previously it has been shown that a diminution in cartilage volume predates radiographic joint space narrowing [1]. We found that an increased BMI was associated with reduced femoral head cartilage volume for women. As BMI is an indirect and surrogate measure that cannot discriminate adipose from non-adipose mass, we also examined the association of body composition and found that measures of adiposity (fat mass and percentage of body fat) were associated with reduced femoral head cartilage volume in women, but not men. In contrast, increased fat-free mass was associated with increased femoral head cartilage volume in men.

This study also found that increased fat mass was associated with an increased risk of prevalent cartilage defects in the central superolateral region of the femoral head for women. There is evidence that the location of cartilage defects within the hip joint may be important, with greater self-reported disability shown to be associated with lesions in the superior location of the hip, a region comparable to our definition of central superolateral [5]. Consistently, we found that in women increased fat mass was associated with an increased risk, while increased fat-free mass was associated with a reduced risk of cartilage defects in the central superolateral but not the central inferomedial region of the femoral head. Even among people with no diagnosed hip OA, cartilage defects are associated with reduced femoral head cartilage volume, a structural hallmark that demarcates people with and without hip OA [24]. Therefore, the results of this study, even in a population with no diagnosed hip OA, likely represent very early structural joint damage.

The mechanisms by which an increased BMI and fat mass adversely affects hip cartilage is unknown. It is possible that deleterious structural changes may in part be due to excessive loading of the hip joint caused by increased body mass. For instance, through altered joint biomechanics, obesity may remodel hip bone. In turn, abnormal bone geometry could act as an intermediary between obesity and cartilage damage. It is well-established that people with abnormal hip bone shape (for example, femoroacetabular impingement) have greater cartilage damage than healthy controls [25]. Clarifying the role of bone geometry as a potential intermediate step is complex as there are a number of different measures that may be used to assess hip bone shape. This was highlighted in a recent review discussing that there is accumulating evidence that the aetiology of hip OA may be due to more subtle abnormalities of the proximal femur and acetabulum [26]. As there may be gender differences in hip bone shape, we have presented gender-specific analyses to deal with any such differences. Acetabular over-coverage (pincer deformity), which is more common in women than men [27], may be one mechanism mediating the association between obesity/adiposity and cartilage damage in women. Nevertheless, whether the central superolateral region of the hip joint is vulnerable to biomechanical damage, such as that imparted by added loading from obesity, is speculative but there is evidence that the effect of obesity on OA cannot simply be explained by mechanical loading. For example, it has long been recognized that obesity is a risk factor for hand OA [28]. Furthermore, adipose tissue that was previously considered to be a passive store of energy is now recognised as a highly metabolic organ releasing various pro-inflammatory cytokines including tumour necrosis factor alpha and interleukin-1, both of which have been postulated to play a key role in cartilage destruction in OA [29,30]. Thus, clarifying the relative contribution of joint loading and meta-inflammation in obesity will be important in optimizing early prevention and treatment of hip OA.

In contrast to fat mass, muscle mass has been shown to be protective against cartilage loss at the knee [31]. Until now, no study has examined similar relationships between body composition and hip cartilage properties. This study has shown that increased fat-free mass is associated with a reduced risk of prevalent hip cartilage defects in women and with increased femoral head cartilage volume in men. It may be that increased muscle mass promotes joint stability and protects against deleterious cartilage changes. Nevertheless, this study has only examined total fat-free mass and has not investigated local muscle mass.

Moreover, an important observation of this study was that the associations between fat mass and cartilage change were significant for women, but not for men. This will need to be confirmed by larger studies but suggests that the influence of BMI and body composition on cartilage is weaker for men than women. This may be partly attributable to the lower percentage of body fat observed in men, as well as the smaller sample of men in this series. However, our data may also support the idea that there are gender differences in risk factors for OA. Previous studies at the knee have demonstrated a similar gender disparity, whereby adiposity measures have been shown to be associated with cartilage pathology in women only [19,20,32]. Hormonal influences may be important in explaining potential gender differences, although the average age of the women at the time of MRI assessment in this study was 67.2 years. Thus it is likely that the women in this study were postmenopausal at the time of MRI, mitigating hormonal differences between women and men of this age. Acetabular over-coverage (pincer deformity), which is more common in women than men [27], may be another mechanism mediating the association between obesity/adiposity and cartilage damage in women. Regardless of the underlying mechanism, these results suggest that gender differences need to be considered in the prevention and treatment of hip OA.

This study has several limitations. A larger study with more men is needed to clarify the gender differences in the relationships between obesity and body composition measures and femoral head cartilage properties. Moreover, radiographs were not performed in this study. Some subjects may have had early radiographic OA. On the other hand, MRI measurement of hip cartilage volume is sensitive and correlates with radiographic hip OA [1], likely attenuating any influence that radiographic disease may have had. Additionally, we recruited a sample with no diagnosis of hip OA. Although we did not perform any clinical assessment, we found that the WOMAC pain index median score was very low (19 for men and 22 for women, out of a total possible of 500), providing further evidence to support that this was a population without significant hip pain. Additionally, obesity and body composition measures preceded cartilage assessment by an average of 16.9 years in this study. This is a strength of the study, given that the exposure (body composition or obesity measures) preceded assessment of structural damage. It is unlikely that there is reverse causation whereby deleterious changes in hip cartilage affects body composition, as this was a sample of individuals without significant hip pain with presumably no activity limitations that may have predated obesity and adiposity. Moreover in healthy populations, measures of obesity and adiposity remain stable. We confirm this by demonstrating a strong correlation between BMI at study inception (1990 to 1994) and when MRI was performed an average of 16.9 years later (*r* = 0.86, *P* <0.0001). Nevertheless, BMI does not capture body composition changes that may occur with ageing and future studies with longitudinal body composition data are required. It has been demonstrated that whole body fat mass remains stable with ageing [33], supporting our contention that adiposity will likely remain stable with the passage of time in a healthy cohort such as ours, and that the likely biggest confounder to this may be age. We have adjusted for age in all our multivariate analyses. While the effect of a one-unit (kgm^−2^) increase in BMI appears to be associated with only a modest reduction in femoral head cartilage volume (26 mm^3^) in women, the mean femoral head cartilage volume in women was 2867 mm^3^. This approximates a 1% (95% CI −1.6% to −0.2%) reduction in femoral head cartilage volume with every unit increase in the BMI, so that a five-unit increase in BMI is associated with approximately a 5% (95% CI −8% to −1%) reduction in femoral head cartilage volume, independent of other risk factors. It has previously been shown that approximately 10% of cartilage volume is lost prior to radiographic joint space narrowing [1]. Subsequently, small increases in BMI are likely to be a major determinant mediating the associated risk for hip OA with obesity. Furthermore, although we found no statistically significant interaction between age and either fat or fat-free mass and femoral head cartilage volume, much larger studies would be needed to exclude this as it may be that the effects of measures of body composition differ in younger compared to older people. Finally, it has been notoriously difficult in epidemiological studies to assess structural changes at the hip joint using MRI. Our division of the anterior, central and posterior regions was adapted from methods used by previously published works with smaller sample sizes [5,6] but these previous works provided no prevalence data of regional structural abnormalities for comparative purposes. We have noted a low prevalence of cartilage defects in the anterior and posterior regions of the femoral head, and larger studies may be needed to overcome this issue at the anterior and posterior femoral head. Our approach has provided the first evidence documenting the importance of the anatomical distribution of cartilage defects and their relationships with body composition measures in the central superolateral region of the femoral head.

## Conclusions

We have shown that increased fat mass was associated with adverse hip cartilage changes in women (reduced cartilage volume and increased cartilage defects), while increased fat-free mass was associated with beneficial cartilage changes in both genders (reduced cartilage defects in the central superolateral region of the femoral head in women; increased femoral head cartilage volume in men). Further work is required to determine whether modifying body composition alters the natural history of hip OA. Preserving or increasing fat-free mass and reducing fat mass may help to reduce the incidence and progression of hip OA.

## Abbreviations

BMI: body mass index
BML: bone marrow lesion
CV: coefficient of variation
ICC: intraclass correlation coefficient
MCCS: Melbourne collaborative cohort study
MRI: magnetic resonance imaging
OA: osteoarthritis
OR: odds ratio
WOMAC: Western Ontario and McMaster University osteoarthritis index
